The article "ZFP36 Binds With PRC1 to Inhibit Tumor Growth and Increase 5-Fu Chemosensitivity of Hepatocellular Carcinoma" was retracted in 2025. Reasons: duplicated images; duplicated data; overlap with earlier publications; concerns about the data.

# ZFP36 Binds With PRC1 to Inhibit Tumor Growth and Increase 5-Fu Chemosensitivity of Hepatocellular Carcinoma

**DOI:** 10.3389/fmolb.2020.00126

**Published:** 2020-07-14

**Authors:** Weiqian Chen, Minjiang Chen, Zhongwei Zhao, Qiaoyou Weng, Jingjing Song, Shiji Fang, Xulu Wu, Hailin Wang, Dengke Zhang, Weibin Yang, Zufei Wang, Min Xu, Jiansong Ji

**Affiliations:** ^1^Zhejiang Provincial Key Laboratory of Imaging Diagnosis and Minimally Invasive Intervention Research, Lishui Hospital of Zhejiang University, The Fifth Affiliated Hospital of Wenzhou Medical University, Lishui, China; ^2^Department of Radiology, Lishui Hospital of Zhejiang University, The Fifth Affiliated Hospital of Wenzhou Medical University, Lishui, China

**Keywords:** hepatocellular carcinoma, ZFP36, PRC1, 5-Fu, migration, invasion

## Abstract

Hepatocellular carcinoma (HCC) is the fifth common cause of tumor-related death worldwide. ZFP36, a RNA-binding protein, decreases in many cancers and its role in HCC remains unclear. This study aimed to investigate the underlying mechanisms by which ZFP36 inhibited HCC progression and increased fluorouracil (5-Fu) sensitivity. We found that ZFP36 was downregulated and PRC1 was upregulated in HCC tissues compared with adjacent non-tumor tissues. *In vitro* investigation presented that ZFP36 acted as a tumor suppressor, while overexpression of PRC1 increased cell proliferation, colony formation and invasion. Further investigations demonstrated that overexpression of ZFP36 inhibited tumor growth and promoted 5-Fu sensitivity in xenograft tumor mice model, which could be reversed when PRC1 overexpressed simultaneously. Luciferase reporter assays and Ribonucleoprotein immunoprecipitation analysis indicated that ZFP36 could bind to adenylate uridylate-rich elements located in PRC1 mRNA 3′UTR to downregulate PRC1 expression. Taken together, our findings identified that ZFP36 regulated PRC1 to exert anti-tumor effect, which suggested a potential therapeutic strategy for treating HCC by exploiting ZFP36/PRC1 axis.

## Introduction

The epithelial–mesenchymal transition (EMT) is a process used during normal wound healing and stem cell regulation that is also synonymous with the progression of cancer (Lamouille et al., 2014). The induction of motile mesenchymal cells is initiated by the dissolution of epithelial cell–cell junctions followed by a change of cellular polarity and the reorganization of the cytoskeleton (Kalluri and Weinberg, 2009). Consequently, the expression of epithelial-related genes is downregulated in preference to an increased expression of mesenchymal specific genes (Sanchez-Tillo et al., 2012; Skalamera et al., 2016). The initial gene expression changes contributing to EMT have been found to involve SNAIL, TWIST, and ZEB (Peinado et al., 2007).

The article "ZFP36 Binds With PRC1 to Inhibit Tumor Growth and Increase 5-Fu Chemosensitivity of Hepatocellular Carcinoma" was retracted in 2025. Reasons: duplicated images; duplicated data; overlap with earlier publications; concerns about the data.

ZFP36, also known as tristetraprolin, is an RNA-binding protein (RBP) which is believed to induce a mesenchymal to epithelial phenotype through the downregulation of TWIST1 and SNAI1 (Yoon et al., 2016). The loss of E-cadherin, which is expressed at high levels in epithelial cells, is considered fundamental to the progression of EMT (Beavon, 2000). Several publications have demonstrated that ZFP36 is linked to cancer thanks to evidence showing its down-regulated state in several tumors (Sanduja et al., 2012; Griseri and Pages, 2014; Montorsi et al., 2016). Interestingly, a very recent paper discovered that ZFP36 deletion could exert anti-tumorigenicity actions due to effects on inflammation and metabolism in a diethylnitrosamine (DEN) hepatocarcinogenesis model (Krohler et al., 2019). But during hepatic tumor progression, ZFP36 acted as tumor-suppressor by inhibiting cell proliferation and migration, and slightly increasing chemosensitivity to doxorubicin and sorafénib (Krohler et al., 2019). However, the underlying molecular mechanism by which ZFP36 inhibits tumor growth in HCC progression remains unclear.

The changes in mRNA stability are ultimately reflected at the protein level in most cells. And the stability of mRNAs can be determined by adenylate uridylate-rich elements (AREs) located in the 3′UTRs that improve the degradation of mRNA (Palanisamy et al., 2012). Thus, AREs are involved in the transient expression of genes that regulate functions associated with cell proliferation, apoptosis, cytokine response, and cellular motility (Bakheet et al., 2001). The basic motifs of which the AREs are composed include pentamers of AUUUA, nonamers of UUAUUUAUU, together with composition of linked pentamers and/or nonamers (Wilusz et al., 2001). The abnormal post-translational control of mRNAs containing AREs is believed to participate in processes that lead to carcinogenesis (Khabar, 2014), since AREs facilitate the binding between RBPs and mRNAs. HuR is an RBP that is abundant in cancer cells and is associated with chemoresistance (Blanco et al., 2016). Poor survival in breast cancer patients is significantly associated with a low ZFP36/HuR mRNA ratio (Hitti et al., 2016).

Protein regulator of cytokinesis 1 (PRC1), is a microtubule-associated protein (MAP) which is involved in cytokinesis and is known to play an important role in the malignant progression of tumors and resistance to chemotherapeutic drugs (Jiang et al., 1998; Shimo et al., 2007; Subramanian et al., 2010; Chen et al., 2016). As a ARE-mRNA that consists of UUAUUUAUU motif, PRC1 has been found over-represented in several cancers, including HCC (Wang et al., 2017; Zhan et al., 2017) and is negatively correlated with a low ZFP36 and human antigen R (HuR, also known as ELAVL1) ratio (Al-Souhibani et al., 2010; Hitti et al., 2016).

The article "ZFP36 Binds With PRC1 to Inhibit Tumor Growth and Increase 5-Fu Chemosensitivity of Hepatocellular Carcinoma" was retracted in 2025. Reasons: duplicated images; duplicated data; overlap with earlier publications; concerns about the data.

In this study, we hypothesized ZFP36 could bind with PRC1 to inhibit tumor growth and 5-Fu resistance in HCC progression. Hence, the role of both ZFP36 and PRC1, and their relationship in regulating were investigated using cell lines as well as the nude mouse model.

## Methods

### Cell Cultures and Reagents

Human hepatoma Huh7, HepG2, SNU475, and Hep3B cells were obtained from Shanghai Institute of Cell Biology, Chinese Academy of Sciences (Shanghai, China). HCC cell lines and normal liver cells (LO2) were maintained in Dulbecco's modified Eagle's medium (Invitrogen, Carlsbad, CA, USA) supplemented with 10% fetal bovine serum (FBS) at 37°C in a humidified atmosphere with 5% CO_2_. 5-Fu was purchased from Sigma-Aldrich (St. Louis, MI, USA). The drugs were stored as 10 mM stock solutions in sterile PBS at −20°C.

### Patients and Tissue Samples

Matched hepatocellular carcinoma and adjacent normal tissue (non- tumor) were acquired from 35 patients who had primary surgical resection at the Lishui Central Hospital (Zhejiang, China). This study was approved by the Ethics Committee of the Lishui Central Hospital of Zhejiang University in accordance with the Declaration of Helsinki and all patients signed informed-consent documents.

### Tissue Microarray Generation and Immunohistochemical Analysis

The construction of tissue microarray (TMA) containing 68 primary HCC and 60 adjacent non-cancerous liver tissues, with the age of the donors ranging between 18 and 73 years (mean age, 48.31 years) was in collaboration with the Shanghai Biochip Company Ltd., Shanghai, China) as described previously (Dong et al., 2017). Immunohistochemistry (IHC) was performed using antibodies (ab51248, 1:500) directed toward PRC1. The positive cell percentage of the immunoreactive staining was classified as 0 (0–4%), 1 (5–24%), 2 (25–49%), 3 (50–74%), 4 (75–100%) and the intensity was scored as 0 (unstained), 1 (light yellow), 2 (brown), 3 (reddish brown). The sum of positive staining was used to define expression levels.

### Construction of Lentiviral Vectors and Stable Cell Lines

To knockdown ZFP36, three short hairpin RNA (shRNA) constructs targeting ZFP36 (ZFP36-shRNA1#, 5′-CGACATAGCTCAGTCTTGTAG-3′; shRNA2#, 5′-AAACAGAGATGCGATTGAAGA-3′; shRNA3#, 5′-GTCAGATCCATGGTGTAACGG−3′); To knockdown PRC1, three shRNAs constructs targeting PRC1 (PRC1-shRNA1#, 5′-TTCAGTTGTCTTTCCTGCTTG-3′; PRC1-shRNA2#, 5′-TTTCCTGCTTGGCTCTCTCTT-3′; PRC1-shRNA3#, 5′-TTGTTCTTCAGTTGTCTTTCC-3′); and a scrambled negative control shRNA (scr, 5′-GACCTGTACGCCAACACAGTG-3′) were chemically synthesized at Genechem (Shanghai, China). The shRNAs were cloned into the PLKO.1-puro recombinant shRNA expression vector (Invitrogen) and co-transfected with the lentiviral packaging helper plasmids, pCMV-dR8.91 and envelope VSV-G (Addgen, Cambridge, MA, USA) into 293T cells using Lipofectamine 2000 (Invitrogen). The supernatants were collected after transfection and concentrated by ultracentrifugation for 72 h. Infected cells were selected by 4 μg/ml puromycin (Invitrogen) for 2 weeks to generate stable cell line.

The article "ZFP36 Binds With PRC1 to Inhibit Tumor Growth and Increase 5-Fu Chemosensitivity of Hepatocellular Carcinoma" was retracted in 2025. Reasons: duplicated images; duplicated data; overlap with earlier publications; concerns about the data.

To overexpress ZFP36 (ZFP36-OE) or PRC1 (PRC1-OE), full length human ZFP36 or PRC1 cDNA was amplified and cloned into the pCDH-CMV-MCS-Puro expression vector and the pCDHpPACKH1TM Lentivector Packaging Kit (System Biosciences, Mountain View, CA, USA) was used to produce lentivirus particles. Infected cells were selected by 4 μg/ml puromycin for 2 weeks to generate stable cell lines.

### Half Maximal Inhibitory Concentration (IC50) Assay

IC_50_ values were the dose required to inhibit the 5-Fu activity of 50% of the cell population and calculated from logarithmic sigmoidal dose-response curves generated using GraphPad Prism 5.0 software (GraphPad Inc). Huh7 and HepG2 cells were grown with 0, 5, 10, 25, 50, 100, 200, and 400 μg/ml of 5-Fu for 7 days.

### Colony Formation Assay

Huh7 and HepG2 cells transfected with vectors were seeded in 6-well plates (300 cells/well) and allowed to attach for 24 h. Cells were grown for 14 days with or without 135 μg/ml 5-Fu for Huh7 cells or 110 μg/ml 5-Fu for HepG2 cells. Colonies were fixed with 4% paraformaldehyde for 60 min and then washed twice by PBS. Finally, colonies were stained with 0.1% crystal violet in 100% ethanol and then counted.

### qRT-PCR

Total RNA was extracted from cultured cells or tissues using TRIZOL reagent (Invitrogen), according to the manufacturer's instructions. Total RNA was reverse transcribed using a PrimeScript RT reagent kit (TaKaRa, Dalian, China) and SYBR Premix Ex Taq II (TaKaRa) according to the manufacturer's instructions. The PCR conditions were carried out using an ABI 7500 real-time PCR system (Applied Biosystems, Foster City, CA, USA). The primers were as follows: ZFP36 forward: 5′-CCCAAATACAAGACGGAACT-3′, reverse: 5′-GCTCTGGCGAAGCACA-3′; PRC1 forward: 5′-GAGTTGAAGGCACGAA-3′, reverse: 5′-TGCATCTCCCATTGTT−3′; Data were normalized to β-actin. The relative quantification of expression was calculated using the 2^−ΔΔCT^ method (VanGuilder et al., 2008).

### Western Blotting

Equal quantities of protein were resolved using 10–15% sodium dodecyl sulfate-polyacrylamide gel electrophoresis and transferred onto polyvinylidene difluoride membranes (Millipore Corporation, Bedford, MA, USA). Membranes were blocked and then incubated with primary antibodies overnight at 4°C. The primary antibodies were ZFP36 antibody (ab33058, 1:500 dilution), PRC1 (ab51248, 1:500 dilution), E-cadherin (ab40772, 1:1000 dilution), N-cadherin (ab18203, 1:1000 dilution), and Vimentin (ab92547, 1:1000 dilution) (Abcam, Austin, TX, USA). Following three 5-min washes in TBS containing Tween20, the membrane was probed with secondary antibody, goat anti-rabbit IgG-HRP (ab6721, 1:10,000) at room temperature for 2 h. After further washing in TBST, immunolabeling was detected using Pierce ECL Western Blotting Substrate (Pierce Biotechnology, Rockford, IL, USA). β-actin was included as a control and densitometric analysis was performed to determine the relative expression of the target proteins.

The article "ZFP36 Binds With PRC1 to Inhibit Tumor Growth and Increase 5-Fu Chemosensitivity of Hepatocellular Carcinoma" was retracted in 2025. Reasons: duplicated images; duplicated data; overlap with earlier publications; concerns about the data.

### Cell Proliferation Assay

Cell proliferation was quantified using a cell counting kit-8 (CCK-8, Dojindo, Kumamoto, Japan) according to the manufacturer's instructions. Briefly, 2,000 cells/well were seeded into 96-well plates and cultured overnight. Cell proliferation was detected at 1–5 days by adding 10 μl CCK-8 reagent and measuring the reaction at A_450nm_ with an Epoch Microplate spectrophotometer (BioTek, Winooski, VT, USA).

### Migration and Invasion

For migration and invasion assays, Huh7 and HepG2 cells were seeded onto uncoated or coated Matrigel in plates with 24-well inserts (BD Bioscience, Bedford, MA, USA). The cells (2 × 10^4^ cells/well in 100 μL serum-free medium) were added to the upper chamber and 600 μL 10% FBS serum medium was added to the lower chamber as a chemoattractant. After 16 h incubation, non-migrating cells were removed by wiping the upper chamber with a cotton swab and migrated cells in the lower chamber were quantified in five random fields using a Nikon microscope at 200 × magnification.

### Tumor Xenograft Model and Tumor Growth Assay

A xenograft tumor model was generated as previously described (Dong et al., 2017). Nude male BALB/cA-nu mice (6-weeks-old) were obtained from the Shanghai SLAC Laboratory Animal Co., Ltd. (Shanghai, China; *n* = 6 per group) and were weighed, coded and randomly assigned to experimental groups. HepG2 cells (2 × 10^6^) were infected with negative control (NC) or ZFP36-OE for ZFP36 overexpression. Infected cells were subcutaneously injected into the flanks of 6-week-old male nude mice to induce tumor formation. Tumor diameters were measured at regular intervals, and the tumor volume was measured every 3 days using the following formula: volume = length × width^2^/2. Mice were sacrificed 27 days after injection and tumor grafts were excised, weighed, harvested, fixed, and embedded for histological examination. All experiments were approved and performed according to the guidelines of the Ethics Committee of Shanghai 10 People's Hospital of China (Shanghai, China), and conformed to the Principles of Laboratory Animal Care (National Society for Medical Research) and were conducted according to the National Institutes of Health guidelines.

The article "ZFP36 Binds With PRC1 to Inhibit Tumor Growth and Increase 5-Fu Chemosensitivity of Hepatocellular Carcinoma" was retracted in 2025. Reasons: duplicated images; duplicated data; overlap with earlier publications; concerns about the data.

### Ribonucleoprotein Immunoprecipitation Analysis

To assess the association of endogenous ZFP36 with endogenous PCR1 mRNA, we performed immunoprecipitation (IP) of ribonucleoprotein (RNP) complexes as described previously (Costantino et al., 2009). Immunoprecipitation was performed using either anti-ZFP36 or immunoglobulin G (IgG) control antibodies. RNA was isolated from the immunoprecipitation, and PRC1 levels of mRNA in ZFP36 IP or IgG IP materials were measured by QRT-PCR in Huh7 and HepG2 cells.

### Luciferase Reporter Assays

Two hundred ninety-three cells were first plated at a density of 50,000 cells/well the day before transfection in 24-wells plates. 3′-UTR cDNA fragments of PRC1 containing the putative wildtype or mutant ZFP36 binding sites were amplified using the following primers: wild type 3′-UTR of PRC1, forward: 5′- CGCCTCGAGCGCCCTCTTTACCTATCC−3′ and reverse: 5′- CGGGCGGCCGCATGAGTAAACAGCGTGGC-3′; mutant 3′-UTR of PRC1 forward: 5′- CGCCTCGAGGAAGCACTATTTAAAATTC−3′ and reverse: 5′- CGGGCGGCCGCGTATGAGTAAACAGCGTG-3′; The amplified cDNA fragments were subcloned into the psiCHECK-2 vector (Promega, USA) at the *Xho*I and *Not*I sites downstream of the luciferase gene. Two hundred ninety-three cells were co-transfected with the luciferase reporter systems and pcDNA3.1-NC or pCDNA3.1-ZFP36 as indicated in figure legends. At 48 h post- transfection, luciferase activities were measured using a Dual-Luciferase Reporter Assay System (Promega) and normalized to Renilla luciferase activity. All experiments were performed in triplicate.

### Immunofluorescence Staining

Cells were grown on glass coverslips, fixed in formalin, rinsed in PBS, and permeabilized with 0.1% Triton-X. Cells were then incubated with primary antibodies E-cadherin (ab40772, 1:100 dilution) and N-cadherin (ab98952, 1:100 dilution) at 4°C overnight followed by goat anti-rabbit IgG H&L (Cy3®) preadsorbed or goat anti-mouse IgG H&L (FITC). Nuclei were counterstained with DAPI (Sigma-Aldrich). Slides were processed using an Axio Observer microscope (ZEISS) with image processing software.

### Statistical Analysis

Results are presented as the mean ± SD from three independent experiments (biological replicates) performed in triplicate (technical replicates). Student's *t*-test was used to detect significant differences between two groups. Significant differences within multiple groups were examined using one-way ANOVA for repeated measures, followed by Dunnett's Multiple Comparison Test or Bonferroni's Multiple Comparison Test. *p* < 0.05 was considered significant. The Pearson chi-square test was used to analyze the relationship between PRC1 expression and clinicopathological features. Survival curves were generated according to the Kaplan–Meier method and statistical analysis was performed using the Log-rank test. Statistical analysis was performed using SPSS 17.0 software (SPSS, Chicago, IL, USA).

The article "ZFP36 Binds With PRC1 to Inhibit Tumor Growth and Increase 5-Fu Chemosensitivity of Hepatocellular Carcinoma" was retracted in 2025. Reasons: duplicated images; duplicated data; overlap with earlier publications; concerns about the data.

## Results

### ZFP36 Is Downregulated and PRC1 Is Upregulated in Hepatocellular Carcinoma Tissues

ZFP36 was downregulated while PRC1 was upregulated in matched HCC than adjacent normal tissue acquired from 35 patients by qRT-PCR (Figures 1A,B) and western blotting analysis (Figures 1D–F). Furthermore, there was a negative correlation between the level of ZFP36 and PRC1 in tumor tissue (*R* = −0.372, ^**^P < 0.026, Spearman correlation) (Figure 1C, Table 1).

**Figure 1:** The expression of ZFP36 and PRC1 in hepatocellular carcinoma tissues. **(A,B)** ZFP36 and PRC1 expression in 35 paired hepatocellular tumor and adjacent non-tumor tissues analyzed by qRT-PCR (*N* = 35). **(C)** The relationship between ZFP36 expression and PRC1 expression was detected by Spearman correlation analysis (*R* = −0.372, **p < 0.026). **(D)** Six pairs of representative bands of ZFP36 and PRC1 protein expression in hepatocellular carcinoma tissues and adjacent non-tumor tissues analyzed by western blots. **(E,F)** Quantifications of the density of western blots were determined by Image J (*N* = 6). (*p < 0.01, **p < 0.01, ***p < 0.001).

**Table 1:** PRC1 staining and clinicopathological characteristics of 103 hepatocellular carcinoma patients.

	**PRC1**			
**Parameters**	**Low (%)**	**High (%)**	**Total**	***P*-value**
Age (years old)				0.114
<50	17 (16.5)	31 (30.1)	48	
≥50	28 (27.2)	27 (26.2)	55	
Gender				0.793
Female	19 (17.2)	23 (24.7)	42	
Male	26 (25.2)	35 (34.0)	61	
Postoperative chemotherapy				0.071
No	29 (28.2)	27 (26.2)	56	
Yes	16 (15.5)	31 (30.1)	47	
TNM stage				0.018^*^
I	19 (18.4)	11 (10.7)	30	
II	16 (15.5)	22 (21.4)	38	
III	10 (9.7)	25 (24.3)	35	

* *p < 0.05, chi-square test*.

### Overexpression of ZFP36 Inhibits Cell Proliferation, Migration, Invasion, and EMT *in vitro*

To further analyze the involvement of ZFP36 in HCC, we measured its expression in the HCC cell lines HepG2, SNU475, Hep3B, and Huh7 and the normal liver cell line LO2 (Figure 2A). ZFP36 expression was significantly higher in the HepG2 cell lines than the control. Moreover, ZFP36 expression was significantly lower in the Hep3B (*P* < 0.05) and Huh7 (*P* < 0.01) cell lines. To further investigate this variation of expression in HepG2 and Huh7 cells, we knocked down the expression of ZFP36 by RNA interference and measured the effects on cell proliferation in HepG2 cells (Figures 2B–D). Downregulation of ZFP36 in HepG2 cells led to a significant increase in cell growth, cell migration and invasion in HepG2 cells as determined by Transwell assay (Figures 2F,G). Whereas, overexpression of ZFP36 in Huh7 cells significantly reduced cell growth (Figure 2E), and inhibited cell migration and invasion in Huh7 cells. We then assessed EMT in HepG2 cells with ZFP36 downregulated and in Huh7 cells with ZFP36 upregulated. The protein expression of the EMT markers E-cadherin, N-cadherin, and vimentin was detected by western blots (Figures 3A,B). Levels of E-cadherin were reduced in HepG2 cells with ZFP36 downregulated but increased in Huh7 cells with ZFP36 upregulated. The opposite pattern was observed with N-cadherin and vimentin. E-cadherin and N-cadherin expression was also detected by immunofluorescence staining in HepG2 and Huh7 cell, respectively (Figure 3C). N-cadherin levels were highest in HepG2 cells downregulating ZFP36 whereas E-cadherin levels were at the highest level in Huh7 cells overexpressing ZFP36. These results indicate that ZFP36 expression is associated with cell EMT.

The article "ZFP36 Binds With PRC1 to Inhibit Tumor Growth and Increase 5-Fu Chemosensitivity of Hepatocellular Carcinoma" was retracted in 2025. Reasons: duplicated images; duplicated data; overlap with earlier publications; concerns about the data.

**Figure 2:** ZFP36 regulates cell growth and cell migration and invasion. **(A)** qRT-PCR analysis of ZFP36 expression in the hepatocellular carcinoma cell lines HepG2, SNU475, Hep3B, and Huh7 and the normal liver cell line LO2. **(B)** Knockdown of ZFP36 (ZFP36 shRNA1#−3#) in HepG2 cells and qRT-PCR assessment of ZFP36 expression. HepG2 cells were transfected with ZFP36-shRNA1# or shRNA2# and Huh7 cells were transfected with ZFP36-OE for ZFP36 overexpression. **(C)** Overexpression of ZFP36 in Huh7 cells and qRT-PCR assessment of ZFP36 expression. **(D,E)** Cell growth was determined by the CCK-8 assay. **(F,G)** cell migration and invasion were detected by Transwell assay. *p < 0.05, **p < 0.01, ***p < 0.001.

**Figure 3:** ZFP36 regulates cell epithelial–mesenchymal transition (EMT). HepG2 cells were transfected with ZFP36-shRNA1# or shRNA2# and Huh7 cells were transfected with ZFP36-OE. **(A,B)** Levels of the EMT markers E-cadherin, N-cadherin and Vimentin were detected by western blots. **(C)** E-cadherin and N-cadherin expression was detected by immunofluorescence staining. *p < 0.05, **p < 0.01, ***p < 0.001.

### Overexpression of ZFP36 Increases Sensitivity to 5-Fu and Decreases Tumor Growth *in vitro* and *in vivo*

We first detected the half maximal inhibitory concentration (IC50) of Huh7 and HepG2 cells treated with serial concentrations of 5-Fu for 7 days (Figures 4A,B). The IC50 of Huh7 cells was 135 μg/ml and for HepG2 cells, it was 110 μg/ml. In a colony formation assay of Huh7 cells, Huh7 overexpressing ZFP36 were more sensitive to 5-Fu than the NC group (Figure 4C). In HepG2 cells, HepG2 with silenced ZFP36 expression exerted less sensitive to 5-Fu than the scr group (Figure 4D).

The article "ZFP36 Binds With PRC1 to Inhibit Tumor Growth and Increase 5-Fu Chemosensitivity of Hepatocellular Carcinoma" was retracted in 2025. Reasons: duplicated images; duplicated data; overlap with earlier publications; concerns about the data.

**Figure 4:** Overexpression of ZFP36 increases sensitivity to 5-Fu treatment *in vitro*. **(A,B)** Huh7 and HepG2 cells were treated with 0, 5, 10, 25, 50, 100, 200, and 400 μg/ml 5-Fu for 7 days, to determine the half maximal inhibitory concentration (IC50). The IC50 of Huh7 cells is 135 μg/ml and the IC50 of HepG2 cells is 110 μg/ml. **(C,D)** A colony formation assay of Huh7 cells transfected with ZFP36 and HepG2 cells transduced with ZFP36 shRNA1# or 2#. Cells were grown for 14 days with or without 135 μg/ml 5-Fu for Huh7 cells or 110 μg/ml 5-Fu for HepG2 cells and stained with crystal violet. The colonies were counted and captured. *p < 0.05, **p < 0.01, ***p < 0.001.

To determine the influence of ZFP36 overexpression on tumorigenicity, tumor growth was assessed in nude mice that were subcutaneously injected in the right flank with either control Huh7 cells or Huh7 cells overexpressing ZFP36. Average tumor weight was measured in mice following treatment with 5-Fu and tumor growth curves were generated (Figures 5A–C). Tumor volume and weight were the lowest in mice who received 5-Fu and Huh7 cells overexpressing ZFP36. However, weight and volume were also significantly reduced in tumors overexpressing ZFP36 without 5-Fu treatment compared to the control. Ki67, ZFP36, and PRC1 expression were detected in tumors by IHC (Figure 5D). Ki67 and PRC1 expression appear to be increased in control cells but levels are reduced in cells treated with 5-Fu. When ZFP36 levels are high, levels of Ki67 and PRC1 are reduced. Taken together, these results indicate that overexpressing ZFP36 increases the overall effect of 5-Fu on tumor growth in nude mice.

**Figure 5:** ZFP36 increases the curative effect of 5-Fu on tumor growth in nude mice. **(A)** The tumor growth curve of ZFP36 overexpressed in Huh7 cells was compared with vector-expressing cells with or without 5-Fu treatment. HepG2 cells (2 × 10^6^) were infected with negative control (NC) or ZFP36-OE. Infected cells were subcutaneously injected into the flanks of 6-week-old male nude mice to induce tumor. Mice were sacrificed 27 days after injection. Photos were captured, and tumor growth was assessed. **(B,C)** Average tumor weight was measured and growth curves were generated. **(D)** Ki67, ZFP36, and PRC1 expression were analyzed by immunohistochemistry (IHC). *p < 0.05, **p < 0.01.

The article "ZFP36 Binds With PRC1 to Inhibit Tumor Growth and Increase 5-Fu Chemosensitivity of Hepatocellular Carcinoma" was retracted in 2025. Reasons: duplicated images; duplicated data; overlap with earlier publications; concerns about the data.

### PRC1 Is Upregulated in Liver Cancer Tissue and Is Associated With a Poor Survival

We used IHC to analyze the expression levels of the PRC1 protein in tissue TMAs of 68 liver cancer tissues and 60 non-tumor tissues (Supplementary Figure 1A). Representative examples of PRC1 staining in high to low grades of cancer tissues are shown in Supplementary Figure 1. The expression of PRC1 appears to be higher in high-grades of HCC tissue. Moreover, there was a significant association between PRC1 expression and the survival of HCC patients (*p* < 0.041, Log-rank test) (Supplementary Figure 1B). The TMAs demonstrate that PRC1 is upregulated in HCC tissue and a high expression of PRC1 is associated with a high-grade of tumor and poor survival. In total 103 HCC patients, no significant differences were found between levels of PRC1 in relation to age, gender or received postoperative chemotherapy. However, the difference in levels of PRC1 between tumor TNM stage was significant (*P* = 0.018) (Table 1).

### Overexpression of PRC1 Increases While Downregulation of ZFP36 Inhibits Cell Proliferation, Migration, and Invasion *in vitro*

To analyze the effects of PRC1 on the regulation of cell growth, cell migration, and invasion, we performed similar experiments to those involving ZFP36. qRT-PCR was used to analyze PRC1 expression in the HCC cell lines HepG2, SNU475, Hep3B, and Huh7 and the normal liver cell line LO2 (Figure 6A). In contrast with the results obtained for ZFP36 (Figure 2A), expression of PRC1 was significantly higher in Huh7 than in HepG2. Silencing PRC1 led to the significantly reduced growth of Huh7 cells (Figures 6B–D) whereas overexpressing PRC1 in HepG2 cells increased cell proliferation, invasion and migration significantly (Figures 6E,F). Silencing PRC1 had the opposite effect, cell invasion and migration were reduced significantly. These results indicate that PRC1 is involved in cell proliferation, migration, and invasion in HCC.

**Figure 6:** PRC1 regulates cell growth, cell migration, and invasion. **(A)** qRT-PCR analysis of PRC1 expression in the hepatocellular carcinoma cell lines HepG2, SNU475, Hep3B, and Huh7 and the normal liver cell line LO2. **(B)** Knockdown of PRC1 (PRC1 shRNA1#−3#) in Huh7 cells and qRT-PCR assessment of PRC1 expression. Huh7 cells were transfected with PRC1-shRNA1# or shRNA2# and HepG2 cells were transfected with PRC1. **(C)** Overexpression of PRC1 in HepG2 cells and qRT-PCR assessment of ZFP36 expression. **(D,E)** Cell growth was determined by a CCK-8 assay. **(F,G)** Cell migration and invasion were detected by Transwell assay, *p < 0.05, **p < 0.01, ***p < 0.001.

The article "ZFP36 Binds With PRC1 to Inhibit Tumor Growth and Increase 5-Fu Chemosensitivity of Hepatocellular Carcinoma" was retracted in 2025. Reasons: duplicated images; duplicated data; overlap with earlier publications; concerns about the data.

### ZFP36 Targets PRC1 mRNA3′ UTR and Regulates PRC1 Expression

We hypothesized that ZFP36 could bind to an ARE in the 3′UTR of PRC1. We mutated the putative ZFP36 binding sites in the PRC1 3′-UTR and co-transfected it with pcDNNA3.1-ZFP36 or a NC into the 293 cell line with a luciferase reporter plasmid containing wild-type or mutant PRC1. Luciferase activity confirmed that ZFP36 cannot bind to the mutated ARE site in the PRC1 3′-UTR (Figures 7A,B). Moreover, IP experiments with RNA–protein complexes from cell lysates using either anti-ZFP36 antibody or control IgG indicate an interaction between endogenous ZFP36 and endogenous PRC1 mRNA (Figures 7C,D). Knockdown of ZFP36 results in an increased level of PRC1 in HepG2 cells whereas the overexpression of ZFP36 in Huh7 cells results in a reduced level of PRC1 protein (Figures 7E,F). These results provide strong evidence that ZFP36 interacts with PRC1 in HCC cells.

**Figure 7:** ZFP36 binds to the PRC1 3′UTR. **(A)** Schematic diagram of the 3′ UTR sequence of PRC1. CR, coding region; UTR, untranslated region, and ARE elements. **(B)** A luciferase reporter plasmid containing wild-type or mutant PRC1 was co-transfected into 293 cells with pcDNNA3.1-ZFP36 or a negative control (NC). Luciferase activity was determined at 48 h after transfection using the dual-luciferase assay and shown as the relative luciferase activity normalized to renilla activity. **(C,D)** Association of endogenous ZFP36 with endogenous PRC1 mRNA. After IP of RNA–protein complexes from cell lysates using either anti-ZFP36 antibody or control IgG, RNA was isolated and used in RT-PCR reactions. PRC1 levels of mRNAs in ZFP36 IP or IgG IP materials as measured by qPCR in Huh7 and HepG2 cells. **(E,F)** Knockdown of ZFP36 (ZFP36 shRNA1#−3#) in HepG2 cells and the overexpression of ZFP36 in Huh7 cells, the protein expression of ZFP36 and PRC1 were detected by western blot analysis. **p < 0.01.

### Sensitivity to 5-Fu by the Overexpression of ZFP36 Depends on PRC1

Finally, we investigate the association between ZFP36 and PRC1 in cell migration, invasion, and sensitivity to 5-Fu treatment. Migration and invasion were reduced in Huh7 cells overexpressing ZFP36 but co-transfected with overexpression of PRC1 counteracted this effect (Figure 8A). In HepG2 cells, the silencing of ZFP36 increased migration and invasion but the simultaneous silencing of PRC1 counteracted these effects (Figure 8B). The sensitivity of Huh7 cells to 5-Fu was greatest when ZFP36 was overexpressed but this sensitivity was reduced by overexpressing PRC1 (Figure 8C). Silencing ZFP36 increased the resistance of HepG2 cells to 5-Fu whereas silencing both ZFP36 and PRC1 increased sensitivity (Figure 8D). These findings indicate that overexpression of ZFP36 decreases cell migration and invasion and increases sensitivity to 5-Fu treatment by the downregulation of PRC1 expression.

The article "ZFP36 Binds With PRC1 to Inhibit Tumor Growth and Increase 5-Fu Chemosensitivity of Hepatocellular Carcinoma" was retracted in 2025. Reasons: duplicated images; duplicated data; overlap with earlier publications; concerns about the data.

**Figure 8:** Overexpression of ZFP36 decreases cell migration and invasion and increases sensitivity to 5-Fu treatment by the downregulation of PRC1 expression. **(A,B)** Huh7 cells were transfected with negative control (NC), ZFP36-OE alone, or co-transfected with ZFP36-OE and PRC1-OE; HepG2 cells were transfected with scr, ZFP36-shRNA2#, or co-transfected with PRC1-shRNA1# or 2# and ZFP36-shRNA2#. Migration and invasion were detected by Transwell assay. **(C,D)** Huh7 cells were transfected with NC, ZFP36-OE alone, or co-transfected with ZFP36-OE and PRC1-OE; HepG2 cells were transfected with scr, ZFP36-shRNA2#, or co-transfected with PRC1-shRNA1# or 2# with ZFP36-shRNA2#; Cells were grown for 14 days with 135 μg/ml 5-Fu for Huh7 cells or 110 μg/ml 5-Fu for HepG2 cells and stained with crystal violet. The colonies were counted and captured. *p < 0.05, **p < 0.01.

## Discussion

Resistance to chemotherapy in liver cancers, such as HCC, is believed to be a synergistic interaction that involves at least 100 different genes, which are stimulated by pharmacological treatment (Tian et al., 2014; Ceballos et al., 2018; Marin et al., 2018). The expression of many of these genes is mediated by ARE-mRNAs and negatively correlated with the ZFP36/HuR mRNA ratio (Hitti et al., 2016). In the present study, we investigated the regulation of PRC1 and its relationship with ZFP36 in resistance to 5-Fu in human hepatoma cell lines.

We found there was a significant difference in the expression levels of ZFP36 and PRC1 between different cell lines. In particular, there was a higher expression of ZFP36 in HepG2 cell lines than in control liver cells whereas expression was significantly lower in the Hep3B and Huh7 cell lines than in the control. Correspondingly, there was a significantly high level of PRC1 in Huh7 cells and lower expression in HepG2 cells. The level of PRC1 expression in the HepG2 and Huh7 cell line is in contrast with the expression of ZFP36. Due to the technological issue that HCC subtypes with ZFP36 overexpressing would have low cell viability, we employed 293T cells to conduct Luciferase reporter assay. The negative correlation involving ARE-mRNA expression and the ZFP36 mRNA expression was verified, which indicated ZFP36 bound with PRC1 via targeting ARE.

The article "ZFP36 Binds With PRC1 to Inhibit Tumor Growth and Increase 5-Fu Chemosensitivity of Hepatocellular Carcinoma" was retracted in 2025. Reasons: duplicated images; duplicated data; overlap with earlier publications; concerns about the data.

The difference in ZFP36 expression levels between the cancer cell lines might be explained by the differential heterogeneity of liver cancer itself (Li and Wang, 2016) and these five cell lines also have rather different phenotypes (Hsu et al., 1993). HepG2 is known to be a well-differentiated cell line therefore perhaps the level of differentiation may be responsible for this factor (Chen et al., 2015). It has been suggested that the expression of ZFP36 in cancer cells is induced by p53 and inhibited by Myc (Rounbehler et al., 2012; Lee et al., 2013). The p53 protein is a transcription factor that is encoded by the tumor suppressor gene TP53 and is associated with genetic repair (Levine and Oren, 2009). A functional p53 is believed to induce cell growth arrest to prevent uncontrolled proliferation and tumor development. It is known that the expression levels of the p53 protein are different in Hep3B, HepG2, and Huh7 cells (Gudkov and Komarova, 2003; Gomes et al., 2015). The p53 protein is not expressed in Hep3B cells but is overexpressed in Huh7 cells and expressed at normal levels in HepG2 cell. Besides, ZFP36 was expressed at a low level in Hep3B cells which are thought to lack p53 expression.

In this study, we demonstrated that a high expression of ZFP36 was able to decrease tumor growth and increase sensitivity to 5-Fu in HCC cells and in a mouse xenograft model. However, high expression of PRC1 increased cell growth, migration, and invasion. Moreover, by overexpressing ZFP36 in a cell line that had a low ZFP36 level, we were able to counteract many tumorigenic characteristics and increase susceptibility to 5-Fu. This reflects the findings of other studies. Montorsi et al. (2016) also found that restoring ZFP36 expression in different colorectal cancer (CRC) cell lines, inhibited EMT and increased susceptibility to anoikis. These authors suggested that ZFP36 downregulation is inversely correlated to the Wnt/β-catenin pathway, which is constitutively activated in CRC, and that there is a loss of posttranscriptional regulatory circuits during tumor development and progression. Coincidently, a recent study also found that overexpressed ZFP36 could decrease EMT and colony formation *in vitro*, and promote chemosensitivity to doxorubicin or sorafenib (Krohler et al., 2019), which further suggested the positive role of ZFP36 in upregulating chemosensitivity of HCC cells. Our work indicated that PRC1 expression is controlled by ZFP36 through ARE-mediated post-translational regulation. Hitti et al. (2016) have discovered that more than 200 ARE-mRNAs correlate negatively with ZFP36 and positively with HuR expression. Among these genes, a cluster of 11 genes, which include PRC1, were found to be important in mitosis, leading the authors to propose that ZFP36 may promote G2–M arrest by fine-tuning the temporal expression of specific ARE-mRNAs.

The article "ZFP36 Binds With PRC1 to Inhibit Tumor Growth and Increase 5-Fu Chemosensitivity of Hepatocellular Carcinoma" was retracted in 2025. Reasons: duplicated images; duplicated data; overlap with earlier publications; concerns about the data.

Whereas the expression of ZFP36 is lower in cancer the expression of HuR is increased (Mazan-Mamczarz et al., 2008). In fact, a ZFP36/HuR ratio exists in cells and is associated with cancer and tumorigenesis in a mechanism that is unclear. ZFP36 functions by mediating the decay of target mRNAs, whereas HuR stabilizes transcripts and promotes the translation of target mRNAs. It is thought that ZFP36 may compete for HuR binding by targeting HuR mRNA (Wang et al., 2016). However, the relationship between ZFP36 and HuR in the regulation of PRC1 has not been involved in our present study. Additionally, ZFP36 and HuR served as RBPs, their regulatory influence on other ARE-mRNAs in HCC progression is not fully understood. More research in this area is warranted to establish the precise molecular mechanism of the ZFP36/HuR association.

To conclude, we were able to confirm that ZFP36 was downregulated and PRC1 was upregulated in HCC tissues compared with adjacent non-tumor tissue. Moreover, a high expression of PRC1 was associated with poor survival whereas high ZFP36 levels were associated with increased survival. Additionally, the overexpression of ZPF36 hinders tumor progression and increases the sensitivity of cells to 5-Fu in a mouse xenograft model, suggesting that ZFP36 may regulate mitosis. Ribonucleoprotein immunoprecipitation analysis and Luciferase reporter assays indicated that ZFP36 may interact with ARE in PRC1 mRNA 3′UTR. Taken together, our findings identified that ZFP36 regulated PRC1 to exert anti-tumor effect, which suggested a potential therapeutic strategy for treating HCC by exploiting ZFP36/PRC1 axis.

## Data Availability Statement

The original contributions presented in the study are included in the article/Supplementary Material, further inquiries can be directed to the corresponding author/s.

## Ethics Statement

The animal study was reviewed and approved by the Affiliated Lishui Hospital of Zhejiang University. Written informed consent was obtained from the individual(s) for the publication of any potentially identifiable images or data included in this article.

## Author Contributions

WC, MC, and ZZ designed research, analyzed data, and wrote the paper. QW, JS, SF, and XW performed experiments and prepared figures. HW, DZ, WY, and ZW advised the design of research, collected the tumor samples, and clinical information. MX and JJ reviewed the paper. All authors read and approved the final manuscript.

## Conflict of Interest

The authors declare that the research was conducted in the absence of any commercial or financial relationships that could be construed as a potential conflict of interest.

The article "ZFP36 Binds With PRC1 to Inhibit Tumor Growth and Increase 5-Fu Chemosensitivity of Hepatocellular Carcinoma" was retracted in 2025. Reasons: duplicated images; duplicated data; overlap with earlier publications; concerns about the data.

## Supplementary Material

Supplementary Figure 1 PRC1 is upregulated in liver cancer tissues. **(A)** Expression levels of PRC1 protein in tissue microarrays (TMAs, 68 paired liver cancer tissues and 60 paired adjacent non-tumor tissues) were determined by immunohistochemistry (IHC). Representative examples of PRC1 staining in cancer tissues and non-tumoral tissues are shown. **(B)** Kaplan–Meier analysis of the relationship between PRC1 expression and survival of hepatocellular carcinoma patients (^*^*p* < 0.041, Log-rank test).

## Abbreviations

PRC1: protein regulator of cytokinesis 1
HCC: hepatocellular carcinoma
EMT: epithelial–mesenchymal transition
5-Fu: 5-fluorouracil
MAP: microtubule-associated protein
ARE: adenylate uridylate-rich elements
HuR: human antigen R
FBS: fetal bovine serum
TMA: tissue microarray
IHC: Immunohistochemistry
CCK-8: cell counting kit-8
IP: immunoprecipitation
RNP: ribonucleoprotein.
